The article "ZeVigilante: Detecting Zero-Day Malware Using Machine Learning and Sandboxing Analysis Techniques" was published in 2022. Journal: Comput Intell Neurosci.

# ZeVigilante: Detecting Zero-Day Malware Using Machine Learning and Sandboxing Analysis Techniques

**DOI:** 10.1155/2022/1615528

**Published:** 2022-05-09

**Authors:** Fahd Alhaidari, Nouran Abu Shaib, Maram Alsafi, Haneen Alharbi, Majd Alawami, Reem Aljindan, Atta-ur Rahman, Rachid Zagrouba

**Affiliations:** ^1^Saudi Aramco Cybersecurity Chair, Dhahran, Saudi Arabia; ^2^Department of Networks and Communications, College of Computer Science and Information Technology (CCSIT), Imam Abdulrahman Bin Faisal University, P.O. Box 1982, Dammam 31441, Saudi Arabia; ^3^Department of Computer Science, College of Computer Science and Information Technology (CCSIT), Imam Abdulrahman Bin Faisal University, P.O. Box 1982, Dammam 31441, Saudi Arabia; ^4^Department of Computer Information Systems, College of Computer Science and Information Technology (CCSIT), Imam Abdulrahman Bin Faisal University, P.O. Box 1982, Dammam 31441, Saudi Arabia

## Abstract

For the enormous growth and the hysterical impact of undocumented malicious software, otherwise known as Zero-Day malware, specialized practices were joined to implement systems capable of detecting these kinds of software to avert possible disastrous consequences. Owing to the nature of developed Zero-Day malware, distinct evasion tactics are used to remain stealth. Hence, there is a need for advance investigations of the methods that can identify such kind of malware. Machine learning (ML) is among the promising techniques for such type of predictions, while the sandbox provides a safe environment for such experiments. After thorough literature review, carefully chosen ML techniques are proposed for the malware detection, under Cuckoo sandboxing (CS) environment. The proposed system is coined as Zero-Day Vigilante (ZeVigilante) to detect the malware considering both static and dynamic analyses. We used adequate datasets for both analyses incorporating sufficient samples in contrast to other studies. Consequently, the processed datasets are used to train and test several ML classiﬁers including Random Forest (RF), Neural Networks (NN), Decision Tree (DT), k-Nearest Neighbor (kNN), Naïve Bayes (NB), and Support Vector Machine (SVM). It is observed that RF achieved the best accuracy for both static and dynamic analyses, 98.21% and 98.92%, respectively.

## 1. Introduction

AV-TEST, the independent research institute for IT security, has witnessed an outburst of malware hitting cyberspace worldwide, involving more than 957.37 million malwares; 17.70 million of them appeared in just September 2019 [1]. Malware is expected to expand further with the emerging cloud applications like the IoT and Big Data. Besides, the promising features provided by the antivirus software are not enough for defeating the tremendous growth of the stealthy malwares, since they outsmart their detection techniques by much enhanced evasive methodologies like self-taught mutations, robustness, and obfuscation. Such malwares have no known signature and therefore are not detectable and the user is not warned of the malware existence before it strikes the system [2, 3]. Hence, due to its growing diversity, variety, and complexity, it becomes a challenging area for research community. Per [4, 5], such attacks are variants of existing malwares that conceal their behavior to escape from detection. Zero-Day malware uses distinct evasion tactics to remain stealth. These tactics are implementable by applying some code tricks like obfuscation and packing. Thereby, detecting them becomes a daunting task. One of the advanced evasion tactics is encrypting the payload with a unique key in each system, mainly the serial number of one of the targeted system devices. There is a pressing need to have an approach that uses analysis and detection to enhance the speed and capacity of the malware classification by including the extracted features alongside the use of ML algorithms to scrutinize it via a sandboxing environment. Thus, the proposed model will help in detecting not only known malware types but also the unknown ones. When analyzing malware, there is a need for an isolated environment for practicing and conducting such analyses. Here comes the usage of sandboxing tools that provide a safe environment to execute and monitor malicious code. Sandboxing is a virtual cage, as it does not allow malicious programs to impact or infect the host operating system or sensitive information [6, 7]. There are different sandboxing environments for analysis such as NORIBEN [8], Sandboxie [9], and Cuckoo sandbox (CS) [10]. Choosing an environment is important as it must be effective and compatible with the proposed model.

The article "ZeVigilante: Detecting Zero-Day Malware Using Machine Learning and Sandboxing Analysis Techniques" was published in 2022. Journal: Comput Intell Neurosci.

For this study, we chose CS as an environment for running malwares and monitoring and extracting their behavior. The choice was based on remarkable advantages of CS in generating automated rich reports in various formats including JSON that can be an ideal input for ML algorithms. The output reports from CS hold valuable information related to the malware execution process including memory dumps for both malware process and machine, network traffics in (PCAP) format, Portable Executable (PE) imports, API calls, and files used or downloaded by the malware. In addition, CS is integrated with diverse platforms which allows the interaction of the users while the malware is executed [10].

The focus of this paper is to extract API call sequences and PE imports using ML algorithms. For malware detection with ML algorithms, the supervised learning approach is used involving two phases: training and testing. In the training phase, the datasets of benign and malware files are fed to one of the ML algorithms after specifying certain values related to the used algorithm to build a predictive model [11]. Besides, examining the built model takes place in the testing phase once the unknown file is processed in the predictive model. Subsequently, the files will be classified on the system, whether they are benign or malware files. In this study, we conducted two different analyses of the executable files, dynamic and static. The dynamic analysis was done by extracting the API call sequences using CS, whereas the static one was done extracting the PE imports section from the CS generated JSON reports. Then, the extracted features were used as an input for the ML algorithms used in this study.

We used the most popular ML algorithms used in binary classification which include Random Forest (RF), Neural Network (NN), Decision Tree (DT), k-Nearest Neighbor (k-NN), Naive Bayes (NB), and Support Vector Machine (SVM). The name of the proposed model, ZeVigilante, is inspired by the two phrases “Zero-Day” and “Vigilante” to imply a framework that has the potentiality of attentively detecting advancing and outsmarting malicious software by sophisticatedly built ZeVigilante for keeping an observant eye on the smartest and most deceptive malwares. ZeVigilante's primary aims and objectives are, first, to enrich the research domain by providing a literature review that presents several techniques and models for detecting and analyzing malware, particularly Zero-Day malware, second, to build and deploy a framework utilizing both ML and sandboxing techniques to analyze executable files and classify them into benign or malware files, providing a model that assists malware specialists and hunters to catch Zero-Day malware, and, finally, to design an enhanced model that results in high accuracy and low false rates in detecting Zero-Day malware.

The rest of the paper is organized as follows: Section 2 presents the related work. The proposed model is described in Section 3. Results are shown in Section 4, and the fifth section concludes the paper.

## 2. Related Work

Approaches for detecting Zero-Day malware have been developed through many research works and articles in the past years. All these applied methods targeted finding machine learning algorithm that achieves highest accuracy with several datasets regardless of the malware analysis they have applied. To monitor and analyze the behavior of the malware and benign samples, CS was used in many models, because it gives the benefit of working on a distributed and scalable sandboxing environment. Many studies have applied and integrated sandboxing and ML techniques. We explored many studies considering the dataset being used and they are presented in Table 1. Studies that used only static features as an input for training and testing the ML models are presented in Table 2. Likewise, the studies that used only dynamic features for the classification are presented in Table 3. Finally, we discussed several studies that used hybrid analysis methods with both static and dynamic features with ML-based approaches as shown in Table 4.

The article "ZeVigilante: Detecting Zero-Day Malware Using Machine Learning and Sandboxing Analysis Techniques" was published in 2022. Journal: Comput Intell Neurosci.

In [14], the authors implemented data extraction, detection, and classification by using Python programming language, while working on preimplemented algorithms from Weka ML toolbox simultaneously. In [29], the authors proposed a detection approach to monitor the behavior of the malware via CS, where it generated an automated report in JSON format containing API calls and some log files to be passed to the next analysis process. To analyze the CS report and memory image, volatility tools were used.

In [10], the authors proposed a detection and classification model of nine malware families, and their suggested solution was in a precise way. Their work includes a behavior analysis for extracting features from API calls to detect any system modifications like registries and mutexes. The extracted features were extremely large; therefore, they used R language to remove the redundant features.

In [17], the authors proposed a scalable architecture for detecting Zero-Day malware through multiple phases, including malware preparation, automated malware analysis, and malware classification. CS is used for automated malware analysis to produce the JSON report. The last phase was implemented at the top of Apache Spark that includes an ML library named MLlib. JSON report is analyzed using Python programming language for extracting malware static and dynamic features. To classify Zero-Day malware, the dataset was trained and labelled using 10-fold cross-validation. RF algorithm achieved the best accuracy and lowest false positive (FP) and false negative (FN) values.

In [20], the authors presented a hybrid novel approach. Using CS environment, they inserted a file to run using dynamic analysis to reveal its malicious intent based on the extracted static information while using several ML algorithms for accuracy evaluation. Three certain labels were defined to show the sample's runtime, which is 20 seconds, 60 seconds, and 300 seconds. As a result, at the end of each run, a JSON report that had a score ranging from 1 to 10 was generated. Using this score, CS classified a file as a malicious one when it is equal to or greater than 5, which meant it was assigned a label of “20 s,” and the file is resubmitted for more analysis for 60 seconds to determine whether CS deems the file as malicious. Next is the 300 seconds if the score does not get a minimum of 5 in which, after that, the decision is made. Moreover, an open-source Python library called SKLEARN is used to implement ML algorithms.

The article "ZeVigilante: Detecting Zero-Day Malware Using Machine Learning and Sandboxing Analysis Techniques" was published in 2022. Journal: Comput Intell Neurosci.

In [28], traditional malware detection systems focus on increasing the accuracy of the malware detection system as they require longer time due to the large set of features; as a result, they are delaying the process of malware detection. The description of various steps involved in the system is as follows: First is the data acquisition, which is to collect samples of malware and valid files. Second is the automated malware analysis, where these samples are used in the CS. Third is the feature extraction, in which, because of JSON report generated by CS, malware features are analyzed, where too many features are obtained. Fourth is the feature selection, in which the related features are filtered through the Information Gain (IG) method, and seven features are selected, which are reliable in the classification process. Fifth is the classification, where this selected feature is used to generate a classification model by using ML algorithm in Weka library. Sixth is the evaluation and validation.

Other works relied on NORIBEN sandboxing, like in [8], where the authors proposed a solution to increase the speed and improve capacity of malware classification by extracting integrated features organized in an Excel format, then converted to CSV format, via static and dynamic analysis using antianalysis techniques through the static stage to extract feature vectors from models: Anti-VM, Anti-Debugging, Suspicious URL Analysis, Packet Analysis, and String extraction. Next is the dynamic phase in which APIs and function calls are extracted from a CSV file that is compatible with Weka using the NORIBEN sandboxing tool. After that, all features extracted from both previous phases are combined to be used in the integrated approach, which ultimately resulted in a better rate detection. The basic phases for building a prediction model are the dataset collection and processing for training and testing the model. Several websites provide malicious datasets for security specialists, forensic analysts, and researchers.

Table 1 presents some dataset information that was used in the previously explored studies on analyzing and predicting malware considering (1) the number of the analyzed benign and malware samples, (2) the analyzed file's types, (3) the families of those malware files, and (4) the resources of those datasets. Based on our exploration for many studies as a part of literature review, the following are the most widely used websites for dataset collection:

1. VirusTotal.com: Scanning engine that aggregates several malware families.
2. Dasmalwerk.eu: A batch of malware varies from adware to bank trojan and beyond like Keylogger and Backdoor.
3. Nothink.org: Holds various Honeypots (*ADB, DNS, SMB, SNMP, SSH, and Telnet*).
4. Virusshare.com: Repository malware samples that provide unpacking feature for the packed malware.
5. Malicia-paper.com: Compromises 11,688 binaries with specifications like the time and the classification of the malware.
6. Kernalmode.info: A forum of reverse engineering and malware analysis. Holds valuable discussions about different malware families.
7. Reversinglabs.com: A website to gain insights into malware files. It provides a platform for automated malware static analysis and has insights on malware topics.
8. Archive.org/details/vxheaven-windows-collection: Windows virus collection.
9. Kaggle.com/malware-classification/data: Dataset of nine families. It has metadata extracted from the file.
10. Zeltser.com/malware-sample-sources: It has several malware dataset websites.
11. Virusign.com: Stores information about the malware like the hash value, size, file type, and virus version.

The article "ZeVigilante: Detecting Zero-Day Malware Using Machine Learning and Sandboxing Analysis Techniques" was published in 2022. Journal: Comput Intell Neurosci.

The schemes in [12, 13, 25] used static analysis, while those in [10, 14, 15] used dynamic analysis for Zero-Day malware prediction. Tables 2–4 enlist the techniques, type of ML algorithms used, the parameters, the extracted features, and the accuracy, respectively, for static, dynamic, and hybrid analyses.

## 3. Proposed Model

Based on the literature review conducted in this study, we found that some studies have used datasets with several samples that are not enough for validating the results such as [21, 22, 26–28], and thus the obtained accuracy of malware detection is not fair to be generalized. Others used only static features to detect malware and we believe relying only on the static features will not enable the trained model to capture the dynamic behavior of the malware, especially when considering the design and nature of Zero-Day malware, like [12, 13, 25]. Moreover, some studies evaluated many ML models with both static and dynamic features but showed low accuracy, such as [8, 16, 20, 24]. Therefore, as a motive, we propose evaluating several ML models for malware detection considering enough samples for both training and testing phases, involving both static and dynamic features, providing a sort of taxonomy on the studies and dataset used for tackling malware detection using ML techniques.

The article "ZeVigilante: Detecting Zero-Day Malware Using Machine Learning and Sandboxing Analysis Techniques" was published in 2022. Journal: Comput Intell Neurosci.

The malware scope of this paper is decided based on the facts and analysis derived previously in which the authors have recommended and nominated these types of malware families that will most probably be analyzed and get closed to Ransomware, Trojans, Backdoors, Spyware, Adware, Botnet, and Obfuscators. Since ZeVigilante executes the targeted files in a controlled environment such as CS to study the behavior of the malware, this paper picked the malicious PE as a feasible file type for the dynamic and the static analysis. PE files are generally running on the Windows platform with .exe extension. PE files provide the required information to the Windows loader on how to manage the executable files. Furthermore, 71.43% of the previous frameworks explained in the literature review have used PE as it has much beneficial metadata that facilitates the feature extraction process and could be a strong indicator of malware. For example, the SizeOfRawData value and the section name indicate the existence of file packing. If the SizeOfRawData is zero, the virtual size will be higher and will be allocated in the memory by the OS, so the malware will unpack the malicious code in that reserved memory space. Besides, the section name examines the most popular utilized packers' names like UPX, ASPack, FSG, and MPRESS. In the execution of the PE malware, several features could be extracted while executing several functions including but not limited to Registries, Packing, Network, Crypto, Memory Manipulation, and Process Creation/Manipulation.

### 3.1. ZeVigilante Components and Interactions

The main components of the proposed framework are the training phase and the implementation and testing phase. The two phases are shown in Figure 1.

*Phase 1: Machine Learning Training*. This phase aims to train ZeVigilante model by learning from the training dataset samples. Since ZeVigilante applies a supervised ML, malware and benign samples must be labelled and inputted into several machine learning algorithms. The model will be trained repeatedly with the same dataset input based on diverse features and parameters for being able to predict on new dataset that has not been seen before based on what it learned in this phase.

*Phase 2: Machine Learning Implementation and Testing*. This phase is to ensure that ZeVigilante provides unbiased evaluation. CS is used for dynamic and static analysis and producing a report containing the dynamic and static features in JSON format. Some of the features are shortlisted to avoid features repetition. The features are input in CSV format to already trained algorithm. The results of the proposed approach are measured by evaluation parameters like accuracy and false positive rate.

The article "ZeVigilante: Detecting Zero-Day Malware Using Machine Learning and Sandboxing Analysis Techniques" was published in 2022. Journal: Comput Intell Neurosci.

### 3.2. ZeVigilante Datasets

In a path of building a comprehended detection system, selecting and preparing datasets are vital. Through the review of the literature, it is discovered that datasets observed, frequently or infrequently, are not well prepared and redrafted to be embedded into proper tools for further investigations of their efficiency in producing high accuracy. In IEEE DataPort, there are several Cuckoo-based correlated datasets, and it is the place where ZeVigilante's dataset has been acquired from. The reason is that dataset in DataPort was found to be preprepared and needs no further correlation; however, it is not perfectly aligned with the objective; thus it needed intensive preprocessing to not only ensure a fully correlated data but also ensure its correctness and genuineness. Based on several searches, two DataPort datasets were picked: Angelo Oliveira's two datasets [30, 31]. The first dataset is the API Call Sequences dataset [30] that holds 42,797 malwares and 1,079 goodwares. It formed a perfect bundle of advantages like providing features as system calls, hashes, and 1 or 0 fields indicating malware or benign, respectively. However, the dataset was immense enough for the hosting machine to deal with due to memory's limited capability, restricting the work to implement filtration technique. Each API call sequence is composed of the first 100 nonrepeated consecutive API calls associated with the parent processes, extracted from the “calls” section of CS's JSON reports. The second dataset, the Top 1000 PE [31] that has more than 40 k files, is a Ph.D. research dataset on malware detection and classification that holds the top 1000 imported functions. This dataset holds several features and is important since it is extracted from CS's PE imports section. Accordingly, VirusShare was referred to for malware samples collection and benign samples were downloaded from the apps and Windows 7 x86 directories.

#### 3.2.1. API Call Sequences Dataset

API Call Sequences dataset offers 307 feature indexes that are numbered from 0 to 306 varying between the name of functions, API calls, and static imports. To support this, JSON reports were produced from CS to check the feature's availability based on generated JSON. In the dataset preprocessing, some filters were applied in Weka like NumericToNominal to turn numeric attributes into nominal ones; this filter was useful after CSV imports to enforce the attributes to become nominal, which helps authors to analyze the results statically and to facilitate its visualizing process. To generate an unpruned decision tree, J48 classifier was applied as a Weka filter with the default confidence threshold for pruning (0.25) with 2 as the minimum number of instances per leaf. In another hand, cost sensitive J48 model was used to solve the issue of the unbalancing between the benign and malware samples. This modification resulted in the following accuracy improvements presented in Table 5.

The article "ZeVigilante: Detecting Zero-Day Malware Using Machine Learning and Sandboxing Analysis Techniques" was published in 2022. Journal: Comput Intell Neurosci.

#### 3.2.2. Top 1000 PE Imports

The Top 1000 PE imports dataset contains both malware and benign samples; it holds 1000 static PE imports, and one of its drawbacks is the unbalancing between the malware and the benign samples. Converting data from numeric to nominal is applied to ease the process of building a trained model, since the data is too large to be processed with available equipment. Similarly, J48 algorithm is used with this dataset to build and evaluate the trained model. To overcome the unbalancing problem, a balancer filter is used where the accuracy of the detection was reduced from 98.9449% to 91.8668%.  Table 6 shows the difference between balanced dataset and unbalanced dataset with J48 model.

### 3.3. Features Selection

Several features could be nominated to analyze the malware files; in this paper, API calls and PE imports are used. API calls are an essential component for programs to be executed, since this is the only way to access the system to continuously establish interactive process. API Call Sequences is used to examine the behavior of a program which can give hints on whether a program being executed is malicious or not based on the calls pattern or sequence, number of calls, and system resources used like memory access and network access. Static and dynamic analysis are means to extract API calls sequence for analysis. PE imports or Portable Executables are generally run with extensions .exe and .dll, where useful information could be extracted from their headers and sections. This work focuses on extracting the imports of the Portable Executables including diverse information like registries, command, process execution, network information, keylogging, cryptographical information, privilege escalation, process, service, and memory manipulation [32–34].  Table 7 shows widely used dynamic and static features.

### 3.4. ZeVigilante Implementation

The goal of this phase is to build a predication model that achieves the highest accuracy based on manipulating the ML parameters and trying several algorithms. The process is presented in Figure 2.

It starts by loading the dataset into algorithms to split it into training and test sets. Afterward, the model is being trained with training dataset and the outcome is a fully trained model. The trained model (prediction model) is evaluated based on test dataset and measured by the prediction accuracy. The whole process is repeated for each algorithm so that each accuracy is correlated with others till the highest accuracy is found. ZeVigilante's analysis interface allows the user to choose between three types of analysis: static, dynamic, and hybrid. For static analysis, the model starts with a user uploading an executable and checking whether it has the .exe extension. Then, the model will calculate file's hash value and run the CS to submit the analysis which takes time between 2 and 3 minutes. Cuckoo's running process will generate a JSON file which the user will upload to the system to perform two steps: (1) extracting the file's features and (2) saving the features in csv format into a user's folder. Afterward, the static analysis will conclude and predict whether the executable's generated JSON file is a malware or not, using the prediction model. In dynamic analysis, ZeVigilante adopts two approaches. The first one is to analyze the files that exist in the testing dataset only to retrieve a valid prediction with algorithms. The second approach uses both CS and machine learning algorithm, which gives a stronger analysis as it accepts analyzing any file desired. It is the same as static analysis except that the feature extraction process is applied with first approach by using file's hash. For the second approach, feature extraction is applied by using the generated JSON report via Cuckoo, and features are saved into user's specified folder as a csv file to be furtherly used in machine learning algorithm prediction process.  Figure 3 presents a flowchart of the hybrid analysis.

The article "ZeVigilante: Detecting Zero-Day Malware Using Machine Learning and Sandboxing Analysis Techniques" was published in 2022. Journal: Comput Intell Neurosci.

## 4. Results and Discussion

Machine learning evaluation parameters settings is a phase where the conduction of confirmation and validation of balanced datasets and acceptable nominated features befall. Moreover, the selection of advantageous requirements can turn ineffectual performance of a learning algorithm into something influential whenever it shows values indicating a proper circumstance of a system's criteria [35–39]. Here, we followed the main commonly used criteria to evaluate different machine learning algorithms on predicting malware. The evaluation criteria are the accuracy, recall, precision, and F1-score based on (1), (2), (3), and (4), respectively [40]. Moreover, we presented the confusion matrix for each experiment.

(1) $$\begin{array}{c} \text{Accuracy}=\frac{\text{Number of correctly predicted samples}}{\text{Total number of all predicted samples}}. \end{array}$$

(2) $$\begin{array}{c} \text{Recall}=\frac{\text{True Positive}}{\text{True Positive}+\text{False Negative}}\text{.} \end{array}$$

(3) $$\begin{array}{c} \text{Precision}=\frac{\text{True Positive}}{\text{True Positive }+\text{False Positive}}. \end{array}$$

(4) $$\begin{array}{c} \text{F}1=2*\frac{\text{Precision}*\text{Recall}}{\text{Precision}+\text{Recall}}. \end{array}$$

We evaluated several commonly used ML methods for malware classification including RF, NN, DT, K-NN, NB, and SVM.  Table 8 shows the detailed results for all the applied ML methods considering the accuracy, precision, recall, F1-score, and mean AUC score. Moreover, Table 9 shows the confusion matrix of both types.

For all analyses, the data for training and testing was split on 70%: 30% basis, respectively. To insure detecting Zero-Day malware, we considered the testing samples to be unseen by the ML models during the training phase.

The highest accuracy of predictions was gained by RF classifier for both PE imports and API call sequences. RF achieved an accuracy of 98.17% with the static dataset and 98.89% with the dynamic dataset. The parameters used for RF are Random_state = 0, n_estimators = 100, and criterion = “entropy.” For the static analysis, the accuracy of RF was low, and it was improved by applying filters like numeric to nominal and attribute selection and tuning RF parameters (n_estimators = 20, random_state = 0) to reach the highest accuracy presented in Table 8. NN recorded a good accuracy of 0.9810 when using the following parameters: solver = “lbfgs”, alpha = 1*e* − 5, and hidden_layer_sizes = (500,500). NN showed better classification of the benign samples than RF, where 64% of the benign samples were classified correctly, while 38% of the benign samples were classified as benign when RF was used. The third tested algorithm was the DT with the following parameters: criterion = “entropy” and the max_depth = 3. The model exhibits better accuracy of 0.985 in the dynamic analysis but it was slightly lower in the static analysis: 0.974. While the static analysis improved when the max_depth was set to 8, the accuracy became 0.976 for the static analysis and 0.986 for the dynamic analysis. The result of the KNN method shown in Table 8 was based on *k* = 100 neighbors. As can be noticed in Table 9, KNN showed the best predication of dynamic analysis, where all malware samples were classified as a malware. Overall, the NB method performed poorly as shown in Table 6. We tried different settings to observe the behavior of the classifier. However, the best accuracy was 56.6% with 9 random states. NB showed very poor result for the static analysis, where 45% of the malware samples were classified as benign. It showed an acceptable classification for the benign samples, because 10% of the benign samples were classified as benign and 90% of them were classified correctly. The SVM method better fits with the static features and gave an accuracy of 0.9756 with linear kernel. SVM implementation implies the following steps: (1) Create object to understand inner processes. (2) Fit a model “slow.” (3) Predicate the value. SVM did not fit the API Call Sequences dataset where it required a lot of the CPU time for training. So, we did not apply it for the dynamic analysis. Generally, it is observed that RF achieved the best accuracy for PE imports and the API call sequence (0.9817 and 0.9889). The process of extracting PE imports from Cuckoo's JSON report reflected a strong classification. So, the framework can address the challenges related to early detection of Zero-Day malware in CS, since it processes the executable files' features in real time with fast and accurate classification.

The article "ZeVigilante: Detecting Zero-Day Malware Using Machine Learning and Sandboxing Analysis Techniques" was published in 2022. Journal: Comput Intell Neurosci.

Further Table 10 shows the obtained accuracy results for both the static and dynamic datasets.

Table 11and Table 12 with Figures 4 and Figure 5 depict the true/false rates (FPR, FNR, TPR, and TNR) [41, 42] for both the static and dynamic datasets, respectively. The lowest FPR for the static dataset is 0.0073 with NB and 0.0084 in the dynamic dataset with DT. Still, RF got the highest accuracy and less than 1% FPR.

### 4.1. Discussion on the Sustainability of Malware Detectors

The sustainability of malware detection techniques is an important factor for measuring the quality of the detectors due to the nature of malware. Retraining the ML-based models with recent datasets requires efforts and time for data collecting, features engineering, preprocessing, and finally training. However, considering the dynamic features of malware, pattern of components communications and the distribution of their accesses improve the capability of ML-based approaches to detect Zero-Day malware.

Several studies highlighted and discussed the sustainability factor when validating malware detectors. In [43], a novel malware detection approach was proposed considering the dynamic characteristics of Android apps as an evolutionary behavior metric used for malware detection and classification. Results showed that such evolution-based malware detection outperformed the benchmarks in the sustainability of malware detection. As an extension to [43], in [44], Cai discussed and evaluated the sustainability metric of malware classifiers as an important validity factor for learning-based classifiers. The sustainability of the classifier refers to the capability of the detection techniques to detect Zero-Day malware using the trained model designed to capture the current malware. For ML classifiers, the sustainability depends on the selected features that result in an enhanced classification considering the evolution of both benign and malware classes. In their study, this has been discussed extensively and then a malware detection approach for Android apps was developed, called DroidSpan, which models the distribution of apps sensitive accesses utilizing a behavior profile of Android apps. The results showed that DroidSpan significantly improved the sustainability compared to the considered baselines in sustainability. Moreover, in [45], the authors proposed a malware detection system for Android, DroidEvolver, considering the sustainability of the detection system so that it can detect the evolution of Android malware. DroidEvolver applied a lightweight update process using online learning techniques with evolving feature set and pseudolabels to generate more reliable detection results. Similarly, in [46], the authors studied the deterioration of learning-based malware detectors for Android apps and the main findings revealed the potential of evolution-based approaches for long-span malware detection. Furthermore, they proposed a new classification approach based on the dynamic behaviors of apps which could capture the pattern of the evolution of malware, hence improving the quality of the learning-based malware detectors.

The article "ZeVigilante: Detecting Zero-Day Malware Using Machine Learning and Sandboxing Analysis Techniques" was published in 2022. Journal: Comput Intell Neurosci.

In our proposed approach, we involved both static and dynamic features for training the ML models toward detecting malware. Regarding the sustainability factor of the proposed approach, there is a need to conduct further experiments considering different time scales of the used samples for both training and testing. This will be considered as an extension to validate the proposed approaches in the future study.

### 4.2. Summary of Contributions

The major findings and contributions of this work can be summarized as follows:

1. One of the recommendations provided by [17] was to incorporate some reduction methods to select the relevant set of features. In the proposed study, this point was considered.
2. Compared with studies presented in the conducted literature review, ZeVigilante used datasets with enough samples for static and dynamic analyses considering variety of malware families. In [25], the authors used dataset with more samples compared to this study; however, their experiments were conducted for only static features obtained from the import section of the files.
3. ZeVigilante achieved a high accuracy, above 96%, with all ML algorithms presented in this study, except NB for static dataset. However, in [27], the authors achieved 100% accuracy by using DT, but the result was biased because they validated their work on 220 samples; therefore, they recommended adding more samples to scale down the infection of the bias influence. ZeVigilante used a huge dataset with variety of malware families. In [25], the recorded accuracy is 99.7%, which is higher than the accuracy recorded by ZeVigilante; however, they considered only the static dataset. Although [28] achieved higher accuracy with 3130 samples (97.9% using RF), our model used larger datasets with more than 40 k samples.
4. In this paper, we conducted a comprehensive literature review on the datasets and approaches involved using machine learning algorithms to detect malware.

The article "ZeVigilante: Detecting Zero-Day Malware Using Machine Learning and Sandboxing Analysis Techniques" was published in 2022. Journal: Comput Intell Neurosci.

## 5. Conclusions

Zero-Day malware is of major concern to the analysts and reverse engineers for the evolving threat and unrestrained expansion mainly due to emerging cloud-based systems [47–50]. In this paper, we introduced ZeVigilante, a framework to detect Zero-Day malware with adoption of ML and sandboxing techniques. The whole deploying and validating process is conducted within the Cuckoo sandbox (CS) environment for a safer progression. Afterward, ZeVigilante is to be considered an integrated system that analyzes executables files considering both static and dynamic analyses to generate reports for users with decisions and results. The main findings and contributions of this study are as follows: (1) providing a detailed literature review that presents several concepts including malware families, features used to classify malware files, datasets that hold benign and malware files, malware analysis techniques, the algorithms, validation and preprocessing, and sandboxing techniques; (2) integrating different ML algorithms (including RF, NN, DT, K-NN, NB, and SVM) with CS by using Python code; (3) extracting the required features including both PE imports and API call sequence from the JSON report and converting the extracted features into a csv file; (4) implementing the proposed framework with interfaces that allow users to conduct experiments and get the validation results of the executable file (malware or a benign). Finally, we depicted the performance of the ML algorithms along with a detailed comparison, where ZeVigilante demonstrated a high accuracy by outperforming most of state-of-the-art approaches. As a future work, for ZeVigilante, dependency on CS imposes limitations on dynamic analysis integration. Thus, it is recommended to build an independent dataset from the CS environment or to build a compatible dataset. Also, the procedure of undergoing static, dynamic, and hybrid analyses at the same time is not very handy, hence building a structure that can expertly undergo one or two analysis types at max based on examination of the executable file uploaded prior to analysis, which will minimize memory load. Moreover, this work is focusing on detecting the malware not classifying it, so a vital improvement on this model is classification. Finally, as discussed in this paper, there is a need to extend this work to include experimental works for evaluating the sustainability metric for the ML-based malware detectors in the future.

The article "ZeVigilante: Detecting Zero-Day Malware Using Machine Learning and Sandboxing Analysis Techniques" was published in 2022. Journal: Comput Intell Neurosci.

## Figures and Tables

**Figure 1:** ZeVigilante structure.

**Figure 2:** Machine learning training and testing flowchart.

**Figure 3:** ZeVigilante hybrid analysis.

**Figure 4:** Static analysis result.

**Figure 5:** Dynamic analysis result.

**Table 1:** Comparative analysis of dataset collection used for malware analysis.

Ref.	Benign	Malware	Families	Resources
[8]	84	25	Mainly consist of adware, spywares, packed malware, and remote administration Trojans	Benign: system directories
				Malware: online sources
[9]	Not mentioned	Not mentioned	Various types: Trojan, spyware, adware, etc.	OpenMalware, softonic
[10]	1156	984	Dridex, Locky, Teslacrypt, Vawtrak, Zeus, DarkComet, CyberGate, Xtreme, CTB-Locker	VirusTotal
[12]	51,223	15,480	Virus, Worm, Rootkit, Backdoor, Constructor, exploit, flooder, Trojan	VX Heavens 2011
[13]	1,800	Not used	Zeus, Carberp, spy-eye, Cidox, Andromeda, DarkConet	C4 security
[14]	Over 270,000	837	Small, OnlineGames, Hupigon, frethog, Zlob	VirusTotal
[15]	4,394	212,505	Sality, Conficker (Downadup), Tidserv, Trojans, fake AV attacks, C & C Bots, failed IM login attempts, Hotbar updates activity	Internet service provider in Asia
[16]	32475	Not mentioned	Hupigon, OnLineGames, Delf, NSAnti, Banker, Zlob, Banload, small, swizzor, Vundo, viru, Lmir, Buzus, farfli, Vapsup, Inject, Zbot, PcClient, fake, and Biforse	VirusTotal
[17]	0.15 million	0.05 million	More than 3000 malware families	VX Heaven
			Including the top 15 families	Nothink
			Tested by: http://www.avg.com	VirusShare
[18]	61,354	17214	Some of them are obfuscated. Trojan, virus, Worm, Rootkit, Backdoor, flooder, and exploit	VirusTotal
[19]	11,688	2,819	Opcode frequencies	Malicia paper
[20]	Not mentioned	Not mentioned	Not mentioned	World's largest malware repository: Reversing Labs, Inc.
[21]	DS1:1408	DS1:454	Not mentioned	Not mentioned
	DS2:2816	DS2:909		
	DS3:4224	DS3:1364		
	DS4:5632	DS4:1819		
	DS5:7040	DS5:2274		
[22]	Dataset 1: 9,339, dataset 2: 15,512	Dataset 1:	Dataset 1: 25 malware families including Trojan, Worm, PWS, Trojan Downloaders	VirusSign
		not mentioned	Dataset 2: 10 families including delf and zbot.	VirusShare
		Dataset 2:		
		not mentioned		
[23]	10,867 from 9 families	1000	Not mentioned	Kaggle Microsoft malware classification challenge
[24]	14,000	14,000	Not mentioned	Malware: VirusShare
				Benign: VIETTEL Corp.
[25]	83,139	84,911	Not mentioned	VirusShare
[26]	5,567	1,174	Backdoor, Rootkit, hoax, Constructor, e-mail worm	Malware: VirusShare

The article "ZeVigilante: Detecting Zero-Day Malware Using Machine Learning and Sandboxing Analysis Techniques" was published in 2022. Journal: Comput Intell Neurosci.

**Table 2:** Comparative analysis of related works with the static analysis.

Ref.	Machine learning	Parameters	Features	Accuracy
[12]	Naïve Bayes (NB)	True positive rate (TPR)	API calls	Not Mentioned
	Sequential Minimal Optimization (SMO) with its four kernels	False positive rate (FPR)		
	Artificial Neural Networks (ANN)	Precision/accuracy		
	J48 Algorithm	Recall		
	k-Nearest Neighbors (kNN)	F-measure		
		ROC area		
[13]	Deep Belief Network (DBN)	Accuracy noise ratio, learning rate, batch size, Rectified Linear, n-gram, Autoencoder	Not Mentioned	Not Mentioned
	Support Vector Machine (SVM)			
[25]	AdaBoost	True positive rate	Pefile (Python module) is used to extract 54 features like SizeOfCode, SizeOfInitializedData, and characteristics: https://pypi.org/paper/pefile/	99.52%
	Bagging	True negative rate		99.72%
	Decision Tree	F-measure		99.50%
	Extra trees	Accuracy		99.76%
	Naïve Bayes	Training time		99.38%
	Gradient Boosting			99.48%
	k-Nearest Neighbors			99.35%
	Logistic Regression			99.41%
	Random forest			99.77%

**Table 3:** Comparative analysis of related works with the dynamic analysis.

Title	Machine learning	Parameters	Features	Accuracy
[10]	Support Vector Machine	True positive rate (TPR)	Behavior analysis: API calls, API address, files,registry keys, mutexes, processes, and DNS queries	94.6%
	J48	False positive rate (FPR)		94.6%
	Naïve Bayes	False negative rate (FNR)		55%
	K-Nearest Neighbor	True negative rate (TNR)		94.6%
	Random Forest	Accuracy		96.8%
[14]	Random Forest	True positive rate	Dynamic features: API calls that consistof strings, registry keys, mutexes, DLLs, etc.	Not mentioned
		False positive rate		
		Positive predictive value		
		F-measure		
		Area under the curve		
[15]	Random Forest	Precision	Network traffic flow analysis	90.96%
	SVM	Recall		42%
	Weighted Linear	F1-measure		50%

**Table 4:** Comparative analysis of related works with hybrid analysis.

Ref.	ML techniques	Parameters	Features	Accuracy
[16]	Naïve Bayes	True positive rate	Signature and dynamic API calls	74.1%
	DT (J48)	False positive rate	CreateWindow[ExA/ExW]	91.1%
	Random Forest	Precision, F-measure, AUC	ExitProcess, ExitThread, GetDiskFreeSpace[A/ExA], etc.	93.02%
[17]	Support Vector Machine	True positive rate	Static features: binary metadata, static import function, packer detection, and sections' information	89.1%
	Naïve Bayes	False positive rate	Dynamic features:	94.0%
	Random Forest	False negative rate, precision, accuracy	API calls, dynamically loaded libraries, dropped files, mutex operation, etc.	98.8%
[18]	Similarity-based machine learning algorithms	Not mentioned	Static features: API system calls, function names and length, Opcodes, segment code, BSS, idata, tls, rdata, reloc, andrsrc. Dynamic features: File system, registry keys, network traffic monitoring, n-grams, and API calls	Not mentioned
[19]	Random Forest	True positive rate	API calls	97.7%
	DT (J48)	False positive rate		100%
	SMO	Precision, accuracy, recall, F-measure		99.5%
[8]	Naïve Bayes	True positive rate	Integrated features: RegDeleteKey, RegOpenKeyEx, GetProcAddress, Loadlibrary, etc.	70.642%
	SVM	False positive rate		60.055%
	Random Forest	Precision, accuracy, recall		73.47%
[21]	Neural Network	Accuracy	Static features: byte, string, PE import, PE metadata. Dynamic features: system calls	92.18%
	Random Forest	Precision		91.70%
	Support Vector Machine	Recall		91.58%
	Decision Tree			89.31%
	k-Nearest Neighbors			88.78%
[22]	Deep Belief Network (DBN)	Accuracy	All PE headers and subleaders	98.8%
		Recall		
	Deep Learning	F-score		
		Precision		
[23]	Dataset 1: Convolutional Neural Network (CNN) + long short-term memory (LSTM)	Accuracy	Static and dynamic features (API calls)	DS1:
	Naïve Bayes, k-Nearest Neighbors	Precision		96.3%
	Random Forest	Recall		80.5%
	Dataset 2:	F1-score		41.8%
	CNN + LSTM			84.3%
	Support Vector Machines			DS2:
	Random Forest, k-Nearest Neighbors			98.8%
	Naïve Bayes			89.2%
				88.4%
				75.8%
				83.7%
[25]	Deep Residual Neural Network	TPR, TNR, FPR, FPR, accuracy	N-gram, entropy histogram (EH), image representation, application programming interfaces (API)	96.24%
[27]	Decision Tree	Accuracy	API calls	97.89%
	Random Forest	Precision		97.54%
	k-Nearest Neighbor	Recall		97.54%
	Extreme Gradient Booting	F1-score		97.54%
[29]	IB1	True positive rate	Integrated features: packer_used, file_size, section_count, susp_sec_count, network_activity, dropped_count, filesread_count, etc.	98.62%
	Naïve Bayes	False positive rate		95.17%
	J48	Precision		99.71%
	Random Forest	F-measure		99.97%
	Bagging	Accuracy		99.65%
	Decision Table			99.78%
	Multilayer Perceptron			97.54%

The article "ZeVigilante: Detecting Zero-Day Malware Using Machine Learning and Sandboxing Analysis Techniques" was published in 2022. Journal: Comput Intell Neurosci.

**Table 5:** J48 model with and without cost sensitivity.

Attributes	Without cost sensitivity	With cost sensitivity
Correctly classified instances	43292 (98.669%)	43172 (98.3955%)
Incorrectly classified instances	584 (1.331%)	704 (1.6045%)
Benign TP	0.637	0.713
Malware TP	0.996	0.991
Benign FP	0.004	0.009
Malware FP	0.363	0.287
Confusion matrix (malware classified as malware)	42605	42403
Confusion matrix (malware classified as benign)	192	394
Confusion matrix (benign classified as benign)	687	769
Confusion matrix (benign classified as malware)	392	310

**Table 6:** J48 model balanced and unbalanced dataset.

Attributes	Without balancing	With balancing
Correctly classified instances	47078 (98.9449%)	43710 (91.8668%)
Incorrectly classified instances	502 (1.0551%)	3869 (8.1332%)
Benign TP	0.994	0.886
Malware TP	0.989	0.951
Benign FP	0.020	0.049
Malware FP	0.006	0.114
Confusion matrix (malware classified as malware)	15314	22621
Confusion matrix (malware classified as benign)	312	1168
Confusion matrix (benign classified as benign)	31764	2700
Confusion matrix (benign classified as malware)	190	21089

**Table 7:** Dynamic and static features.

Feature	Description
DLL	Helps in promoting modularization of code. It is used in the analysis for revealing the malware's behavioral characteristics since executable needs to import/export the dll.
API calls	Examines the behavior of a program which can give hints on whether a program being executed is malicious or not based on the calls pattern or sequence, number of calls, and system resources used like memory access and network access.
Mutexes	Usually, they are used in voiding simultaneous access to a resource.
Registry system activities	Include critical information about the hardware device, installed software, values, and options used by different processes. Malware usually changes multiple registries to bypass the firewall and safety of window and for self-lunching.
Network activities	Distinguishes malicious activities, connection to malicious servers, malicious download, remote control, malicious URLs, IPs, and ports.
File system	Info about the files' modification, creation, deletion, accesses, etc. Malware modifies and uses it for stealing critical information, infecting the system, and leaving backdoors.
Static imports	Provide valuable information about functions coming from libraries. They play a crucial role in giving a basic overview of the binary intent.
Packers	Encrypt and compress the malware. Malware analysts use them for detecting packers' types and for getting more information about the compressing techniques.
Strings	Strings that might indicate the existence of a malware such as cookie data, URLs, messages, or copies of the file at specific location are detected.
PE	Includes valuable info about code, libraries, spaces, time/date, sections, and resources.

**Table 8:** Results of applied ML algorithms.

Classifier	Analysis type	Accuracy	Precision	Recall	F-score	Mean AUC score
RF	Static	0.9817	0.98	0.98	0.98	0.9876
	Dynamic	0.9889	0.99	0.99	0.99	0.9871
NN	Static	0.9810	0.98	0.98	0.98	0.9740
	Dynamic	0.9688	—	—	—	0.6732
DT	Static	0.9754	0.98	0.98	0.97	0.975
	Dynamic	0.9829	0.98	0.98	0.98	0.982
K-NN	Static	0.9644	0.96	0.96	0.96	0.964
	Dynamic	0.9845	0.98	0.98	0.98	0.984
NB	Static	0.5660	0.95	0.75	0.69	0.56
	Dynamic	0.9066	0.96	0.91	0.93	0.90

The article "ZeVigilante: Detecting Zero-Day Malware Using Machine Learning and Sandboxing Analysis Techniques" was published in 2022. Journal: Comput Intell Neurosci.

**Table 9:** Static and dynamic analysis confusion matrix for all used ML.

ML method	Type of features	Confusion matrix		
		Type	Malware classified as…	Benign classified as…
RF	Static analysis	Malware	13661	352
		Benign	48	213
	Dynamic analysis	Malware	12837	140
		Benign	5	181
NN	Static analysis	Malware	13634	199
		Benign	72	369
	Dynamic analysis	Malware	12614	172
		Benign	238	1391
DT	Static analysis	Malware	9043	153
		Benign	81	239
	Dynamic analysis	Malware	8480	72
		Benign	78	146
K-NN	Static analysis	Malware	13501	307
		Benign	200	266
	Dynamic analysis	Malware	12864	211
		Benign	0	88
NB	Static analysis	Malware	7543	56
		Benign	6138	537
	Dynamic analysis	Malware	11787	199
		Benign	1030	147

**Table 10:** Machine learning algorithms' accuracy.

Algorithm	Static dataset	Dynamic dataset
RF	0.9817	0.9889
NN	0.9810	0.9688
DT	0.9754	0.9829
K-NN	0.9644	0.9845
NB	0.5660	0.9066
SVM	0.9756	Not available

**Table 11:** False and true rates result (static dataset).

Algorithm	FPR	FNR	TPR	TNR
RF	0.0169	0.1306	0.8693	0.9830
NN	0.0143	0.1632	0.8367	0.9856
DT	0.0207	0.1988	0.8011	0.9792
K-NN	0.0222	0.4291	0.5708	0.9777
NB	0.0073	0.9195	0.0804	0.9926

**Table 12:** False and true rates result (dynamic dataset).

Algorithm	FPR	FNR	TPR	TNR
RF	0.0107	0.0268	0.9731	0.9892
NN	0.0134	0.6312	0.3687	0.9865
DT	0.0084	0.3482	0.6517	0.9915
K-NN	0.01613	0.0	1.0	0.9838
NB	0.0166	0.8751	0.1248	0.9833

## Data Availability

The datasets used in the study are from previously reported dataset sources, which have been cited. The processed data are available from the corresponding author upon request.
